# An Improved Bearing Fault Diagnosis Model of Variational Mode Decomposition Based on Linked Extension Neural Network

**DOI:** 10.1155/2022/1615676

**Published:** 2022-04-25

**Authors:** Tichun Wang, Jiayun Wang

**Affiliations:** College of Mechanical and Electrical Engineering, Nanjing University of Aeronautics and Astronautics, Nanjing 210016, China

## Abstract

In bearing fault diagnosis, due to the insufficient obtained supervised data and the inevitable noise contained in the vibration signals, the problem of clustering bearing fault diagnosis with imbalanced data containing noise is caused. Thanks to the ability to quickly and fully learn boundary information in small samples, the extension neural network-type 2 algorithm (ENN-2) has the potential in imbalanced data clustering and has been gradually applied in fault diagnosis. Therefore, in order to improve the unstable clustering performance of ENN-2 caused by its heavy dependence on input order of samples, a novel algorithm called linked extension neural network (LENN) is developed by redesigning the correlation function and its iterative method, which greatly reduces the clustering iteration epochs of the algorithm. In addition, an evaluation index of clustering quality for this novel algorithm, extension density, is also proposed. After that, a bearing fault diagnosis model of variational mode decomposition (VMD) based denoising and LENN is proposed. Firstly, VMD is used to get intrinsic mode functions (IMFs), and the correlation coefficients of IMFs are calculated for signal denoising. Secondly, the features are extracted from denoised signals and selected by PCA algorithm, and the fault diagnosis is finally completed by LENN. Compared with ENN-2, K-means, FCM, and DBSCAN based models, the proposed model identifies the faults with different severities more accurately and achieves superior diagnostic ability on different imbalance degrees of datasets, which can further lay a foundation for clustering fault diagnosis based on vibration signals.

## 1. Introduction

Bearing is one of the most common connecting parts in rotating machinery, which is more likely to break down because of wear, fatigue, corrosion, or overload. Therefore, diagnosis timely and accurately of bearing conditions is of great significance to ensure the mechanical operation steady and reliable. Much study in recent years has focused on bearing fault diagnosis based on vibration signals, including signal acquisition and noise reduction, feature extraction and selection, and fault recognition. However, in industry, diagnostic data is often derived from monitoring signals, bringing great difficulties to record the machinery conditions by frequent downtime checking or manual labeling, which is time-consuming and laborious and resulting in insufficient labeled data for fault diagnosis [1]. Moreover, the number of obtained fault samples is always far less than that of normal samples from monitoring signals, generating the diagnostic problem of imbalanced data.

Clustering analysis is especially suitable for fault recognition when there is no sufficient labeled data. Because of the nonlinear and unstable characteristics of bearing vibration signals, scholars preserve in their attempts to construct clustering diagnosis models with stronger identification ability. For example, after processing the data by ensemble empirical mode decomposition (EEMD) and linear discriminant analysis (LDA), Hou et al. [2] used Gath-Geva clustering algorithm (GG) to identify the faults of rolling bearing and got a satisfactory clustering result with better intraclass compactness. Chang et al.[3] achieved 96% accuracy of permanent magnet synchronous motors demagnetization fault diagnosis by auto-encoder and K-means algorithm. In addition, Li et al. [4] integrated K-means in the neural network architecture for unsupervised learning and proposed a deep representation clustering-based diagnosis model to address the data sparsity issue in data-driven machinery fault diagnosis. Also, K-means was utilized together with K-nearest neighbor algorithm (KNN) to identify a transformer's fault category by cumulative votes [5]. On the other hand, for the algorithms which are unnecessary to set the number of fault categories before clustering, the study of Li et al. [6] describes a method to generate clustering template of rolling bearing so as to reduce the effect of noise on diagnostic accuracy using density-based spatial clustering of applications with noise (DBSCAN). This algorithm was also widely used in wind turbine condition monitoring [7] and diagnosis [8], photovoltaic power station fault detection [9], bolts with mission pins on transmission lines detection [10], and thermal runaway diagnosis of battery systems [11]. Moreover, Wei et al.[12] adopted affinity propagation clustering algorithm (AP) and a novel adaptive feature selection technique to identify different fault categories and severities of bearings successfully, and another bearing fault diagnosis model based on expectation maximization algorithm (EM) and wavelet packet was proposed by Zhang et al. [13] for coal cutter. Other clustering algorithms, including spectral clustering [14], fuzzy C-means (FCM) [15], clustering by fast search and find of density peaks algorithm (CFSFDP) [16], and extension neural network-type 2 (ENN-2) algorithm [17–19] were also applied to diagnosis. In conclusion, the clustering algorithms represented by K-means need to know the number of fault categories before clustering, which is contrary to the fact that clustering analysis does not require prior knowledge; however, the clustering algorithms represented by DBSCAN do not need to know the number of fault categories, but suffer a complex parameter adjustment process during training. Therefore, there remains a need for an efficient clustering method with less prior knowledge, simple parameter tuning process, and stable performance.

At the same time, considering the vibration signals used for fault diagnosis not only contain the running state signals of bearings but also contain a lot of aliasing signals with noises, signal denoising methods have generated considerable recent research interest. The commonly used denoising methods mainly include wavelet threshold denoising method, empirical mode decomposition (EMD), ensemble empirical mode decomposition (EEMD), and local mean decomposition (LMD). For example, Komaty et al. [20] introduced a signal-filtering method of EMD and a similarity measure. In their studies, white Gaussian and colored noises were almost removed from the signals by selecting the decomposed modes according to the similarity between the estimation of the probability density function (pdf) of the input signal and that of each mode, and combined EEMD with grey theory, Jia et al. [21] removed the noise of signals by evaluating noise levels of decomposed components of signals by grey relational analysis and selecting the noise-dominant components by grey model. Yang et al. [22] proposed an adaptive signal denoising method based on LMD. However, these decomposition methods have end-effect and modal aliasing phenomena and are more sensitive to sampling frequency, resulting in pretty large decomposition error. To overcome the defects above, Dragomiretskiy and Zosso [23] in 2014 have proposed variational mode decomposition (VMD), which is a new time-frequency analysis method with adaptive signal. Based on VMD, some research combined this method with other algorithms for signal denoising, such as singular value decomposition (SVD) [24], data-driven time-frequency analysis (DDTFA) [25], and wavelet threshold noise reduction [26], and there were also many studies that selected the decomposed modes in some evaluation methods and reconstructed the signal after VMD for noise reduction, such as kurtosis criterion [27], Bhattacharyya distance [28], and a novel parameter called signal clarity proposed by Li et al. [29]. In addition, Wang et al. [30] used VMD innovatively to eliminate outliers and noise points in features extracted from signals so as to achieve the purpose of signal-filtering and denoising.

However, few researchers have addressed the problem of bearing clustering fault diagnosis on imbalanced data with noise at the same time. Thus, in this paper, close attention is paid to develop an effective clustering algorithm on imbalanced data and construct a bearing fault diagnosis model dealing with the insufficient data contained noise. In our study, an improved clustering algorithm of ENN-2, called linked extension neural network (LENN), is proposed firstly, and based on this algorithm and VMD-based denoising method, a novel bearing fault diagnosis model is presented and applied to analyze the fault conditions and severities of bearings. To validate the effectiveness of the proposed algorithm and the model, three comparative experiments are designed and conducted on commonly used artificial clustering datasets and real bearing fault signals. The results manifest that the proposed model yields higher identification accuracy of minority fault clusters on imbalanced data with noise comparing with the models based on ENN-2, K-means, fuzzy C-means (FCM), and DBSCAN. Our study provides a promising method for machinery fault diagnosis based on insufficient labeled signals with imbalance, permitting an easier parameter adjustment process with less prior knowledge.

The rest of this paper starts with the novel LENN algorithm in Section 2.  Section 3 provides a brief description of the proposed model, and the proposed algorithm and model are experimentally verified in Section 4. In Section 5, the concluding remarks are drawn.

## 2. Linked Extension Neural Network

Extension neural network-type 2 algorithm (ENN-2) is a new clustering algorithm based on extension theory [31]. With no need to set the number of clusters manually in advance, ENN-2 shows good clustering ability and fast convergence speed in simple construction. But in fact, the performance of ENN-2 relies heavily on the initial points and correct input order of the samples. To overcome these deficiencies, we develop a novel clustering algorithm called linked extension neural network (LENN).

### 2.1. Network Structure

Following the form of ENN-2, the structure of LENN contains only two layers, which is shown in Figure 1. The number of input layer nodes depends on the feature dimension of data, and the number of output layer nodes is determined by the number of clusters. Between the two layers, the upper and lower bounds of the clusters connect the neurons as the connection weights, and output neurons are successively constructed in the process of iteration (represented by color shades in Figure 1), with only one node activated at a time to indicate the clustering result.

### 2.2. Improved Correlation Function

#### 2.2.1. Correlation Function in ENN-2

In ENN-2, the correlation function ED based on the extension distance is used to measure the distance between a sample and a target cluster. The extension distance in extension theory describes the distance between a point *x* and an interval *V*=〈*a*, *b*〉 quantitatively, which is defined as

(1) $$\begin{array}{c} \rho \left(x,V\right)=\left|x-\frac{a+b}{2}\right|-\frac{a-b}{2}, \end{array}$$

where *a* and *b* are the lower and the upper bounds of *V*, respectively.

Given the center of the *k*th cluster is Z_*k*_=[*z*_*k*1_, *z*_*k*2_, ⋯, *z*_*kn*_], the boundary of the *k*th cluster can be represented by introducing a hyperparameter to measure the distance between the center and the ideal boundary as

(2) $$\begin{array}{c} W_{k}=\left[\langle a_{k1},b_{k1}\rangle ,\langle a_{k2},b_{k2}\rangle ,\ldots ,\langle a_{kn},b_{kn}\rangle \right]\\ =\left[\langle z_{k1}-\lambda ,z_{k1}+\lambda \rangle ,\langle z_{k2}-\lambda ,z_{k2}+\lambda \rangle ,\ldots ,\langle z_{kn}-\lambda ,z_{kn}+\lambda \rangle \right], \end{array}$$

Also, based on the definition of extension distance, the correlation function ED between a sample *X*=[*x*_1_, *x*_2_, ⋯, *x*_*n*_] and the boundary *W*_*k*_ of the *k*th cluster is defined as

(3) $$\begin{array}{c} ED_{k}=\overset{n}{\underset{j=1}{\sum }}\left[\frac{\left|x_{ij}-z_{kj}\right|-\left(b_{kj}-a_{kj}\right)/2}{\left|b_{kj}-a_{kj}\right|/2}\right],\;k=1,2,\ldots ,K. \end{array}$$

As shown in Figure 2, ED measures the extension relationship between a feature and its boundary. From Figure 2, it can be seen that, for the *j*th dimension of the *k*th cluster, when *x*_*j*_ ∈ 〈*a*_*kj*_, *b*_*kj*_〉, *ED*_*kj*_ ≤ 1.

For a sample *X*=[*x*_1_, *x*_2_, ⋯, *x*_*n*_] with *n*-dimensional features, the sample *X* could be classified into the *k*th cluster if

(4) $$\begin{array}{c} ED_{k}\leq n,\;k=1,2,\ldots ,K. \end{array}$$

Thanks to this property of ED, the algorithm can estimate a sample belongs to which cluster and update the boundary and the center of the corresponding cluster to revise its information for iteration. Therefore, ENN-2 does not require the number of clusters *K* before learning and can obtain better clustering results by only adjusting the unique hyperparameter *λ*.

However, since the input order of samples determines the updating direction of clusters' boundaries and centers in the iteration process, ENN-2 is greatly affected by the initial point selection and the input order of samples and shows unstable clustering performances. Therefore, it is necessary to improve this algorithm.

#### 2.2.2. Improved Correlation Function in LENN

Different from ENN-2, each sample could be considered as a center during iteration in LENN. Take *X*=[*x*_11_, *x*_12_, ⋯, *x*_1*n*_] for example, its boundary *W*_*X*1_ can be represented as (4) with the hyperparameter *λ*:

(5) $$\begin{array}{c} W_{X_{1}}=\left[\langle a_{x_{1}1},b_{x_{1}1}\rangle ,\langle a_{x_{1}2},b_{x_{1}2}\rangle ,\ldots ,\langle a_{x_{1}n},b_{x_{1}n}\rangle \right]\\ =\left[\langle x_{1}-\lambda ,x_{1}+\lambda \rangle ,\langle x_{2}-\lambda ,x_{2}+\lambda \rangle ,\ldots ,\langle x_{n}-\lambda ,x_{n}+\lambda \rangle \right]. \end{array}$$

In order to measure the correlation distance between the sample *X*=[*x*_21_, *x*_22_,…, *x*_2*n*_] and *W*_*X*1_, the new correlation function is defined as

(6) $$\begin{array}{c} ED_{X_{1},X_{2}}=\overset{n}{\underset{j=1}{\sum }}\left[\frac{\left|x_{2j}-x_{1j}\right|-\left(b_{x_{1}j}-a_{x_{1}j}\right)/2}{\left(b_{x_{1}j}-a_{x_{1}j}\right)/2}+1\right]\\ =\overset{n}{\underset{j=1}{\sum }}\left[\frac{\left|\left|x_{2j}-x_{1j}\right|\right|}{\lambda }\right]. \end{array}$$

The new correlation function is plotted in Figure 3. For the *j*th feature of the two samples, when *X*_2*j*_ ∈ 〈*a*_*X*_1_*j*_, *b*_*X*_1_*j*_〉, ED_*X*_1_*j*,*X*_2_*j*_ ≤ 1, and taking all features into account, the sample *X*_2_ could be considered to belong to the same cluster as sample *X*_1_ if

(7) $$\begin{array}{c} ED_{X_{1},X_{2}}\leq n. \end{array}$$

### 2.3. Learning Algorithm of LENN

The learning process of LENN is an unsupervised learning. It takes a dataset *X*=[*x*_1_, *x*_2_, ⋯, *x*_*m*_] with samples as the input, and after calculating the correlation distances between samples level by level, the clustering results of the dataset are finally output in just one epoch. The specific learning steps are as follows:

1. Set an optimal hyperparameter *λ* in $\left(0\sqrt{\max\left(x_{ij}\right)}\right]$.
2. Input a sample *X*_*i*_=[*x*_*i*1_, *x*_*i*2_, ⋯, *x*_*im*_] randomly and mark the cluster which belongs to as *k* = 0. Calculate the improved correlation function ED between *X*_*i*_ and all the other unmarked samples according to equation (5) and mark the samples which meet the requirements of ED ≤ *n* as *k*=0. (3) For all the qualified samples in step (2), each sample is taken as the center to traverse, and EDs between this sample and all the remaining unmarked samples are calculated. Similarly, the samples that meet the condition of ED ≤ *n* are also marked as *k*=0 until no qualified samples left. (4) A sample is randomly generated from the remaining unmarked samples for input to create a new cluster *k*=*k*+1. Repeat steps (2) and (3).
3. The learning process is finished until all samples are marked.

At the end of the iteration, if a cluster contains too few samples, it can be regarded as noise.

The iterative approaches of ENN-2 and LENN are both graphically presented in Figure 4. During the iteration, ENN-2 needs to update the central coordinates each time (represented by the orange dots), and the updating direction is significantly affected by the input order of the samples. Ideally, the input order of the samples should be sorted according to the distance between samples from small to large, which is pretty difficult to ensure for the unpretreated messy datasets. As can be seen from Figure 4(a) clearly, sample 6 is closer to the center corresponding to sample 4 than sample 5. If sample 6 is input for calculation first according to (3), the result meets the requirement of (4), indicating sample 6 and samples 1∼4 belong to the same cluster, and then the final clustering results of the whole dataset contain 2 clusters. But, if input sample 5 first for calculation, the result of (3) does not satisfy (4) because of the distant relationship of sample 5 and the current center, and then a new cluster is created for iteration, resulting in the final results of 3 clusters. However, in Figure 4(b) of LENN, one specific sample is regarded as the center each time, and all the qualified samples which satisfy (7) with the sample are found and marked in this iteration. Taking two-dimensional eigenspace as an example, the learning essence of LENN is to find the samples consecutively which fall in the square constructed by the initial center sample with 2*λ* as the side length. All the qualified samples are classified into the same cluster with their center. And then, the next iteration begins with a subsample of the cluster. Finally, all qualified samples of the same cluster are found by this iterative linkage method. Therefore, in Figure 5, samples 1, 4, 6, 5, and 10 are successively taken as the centers for iteration, and the final clustering result contains only 2 clusters with samples 1∼9 belonging to the same cluster.

According to the learning process of the algorithm, LENN has the following remarkable advantages:

1. Based on extension distance, LENN defines a new approach to categorization by distance calculation.
2. There is no need to preset the number of clusters as in ENN-2; in addition, it is not necessary to initialize clustering center.
3. The improved algorithm only needs one epoch to complete the clustering process and converges faster.
4. LENN is not sensitive to the initial center and the input order of the samples and preserves more stable clustering ability than ENN-2.

Nevertheless, LENN is very sensitive to the hyperparameter *λ*, so it is necessary to select the optimal *λ* before learning.

### 2.4. Parameter Selection Method

In LENN, the selection of the hyperparameter *λ* seriously affects the final number of clusters and the accuracy of clustering results. As shown in Figure 5, for a smaller *λ* (such as *λ*  = 7.2 in Figure 5(a)), the constructed squares will be smaller with fewer qualified samples contained, resulting in more clusters in the end, and for a bigger *λ* (such as *λ*  = 8.7 in Figure 5(b)), the constructed squares will be likewise bigger with more qualified samples contained, and fewer clusters are produced finally.

For clustering algorithms, silhouette coefficient is often used for evaluation with no real labels. However, this index is more suitable to analyze the clustering effectiveness of balanced data [32]. Considering this paper is primarily concerned with imbalanced data clustering problem, a novel evaluation index extension density EDe is developed to tune the hyperparameter *λ* based on extension distance, which is defined as

(8) $$\begin{array}{c} E\;De=\overset{C}{\underset{k=1}{\sum }}\frac{\sum_{x_{i}\in M_{k},j=1}^{n}\left|x_{ij}-z_{kj}\right|-b_{kj}-a_{kj}/2}{m_{k}}, \end{array}$$

where *m*_*k*_ is the number of samples in the *k*th cluster, *Z*_*kj*_ is the center of the *j*th feature, and *a*_*kj*_ and *b*_*kj*_ represent the lower and upper bounds of the *k*th cluster respectively, *a*_*kj*_, *b*_*kj*_ and can be computed by

(9) $$\begin{array}{c} a_{kj}=\min_{x_{i}\in M_{k}}\left(x_{j}\right),\\ b_{kj}=\min_{x_{i}\in M_{k}}\left(x_{j}\right),\\ z_{kj}=\frac{b_{kj}-a_{kj}}{2}. \end{array}$$

Typically, EDe declines with the increasing *λ*, and the optimal *λ* lies in the turning point of the curve.

## 3. Proposed Bearing Fault Diagnosis Model

### 3.1. Signal Denoising

Bearing vibration signals tend to present nonlinear and nonstationary characteristics with noise inevitably. Without signal denoising, the outliers in raw data will be transferred into the feature space through feature extraction and affecting the diagnostic results of the model. Compared with empirical mode decomposition (EMD) and ensemble empirical mode decomposition (EEMD), variational mode decomposition (VMD) can effectively extract each frequency component of the signal and solve the problems of mode mixing and white noise. Therefore, VMD-based method is used for noise reduction in this paper.

#### 3.1.1. The Principle of VMD

VMD is a variational problem solving process based on classical Wiener filter, Hilbert transform, and mixing, which can be written as the following constrained optimization form:

(10) $$\begin{array}{c} \underset{\left\{u_{k}\right\},\left\{\omega_{k}\right\}}{\min}\left\{\underset{k}{\sum }{\left\|\partial_{t}\left[\left(\delta \left(t\right)+\frac{j}{\pi t}\right)*u_{k}\left(t\right)\right]e^{-j\omega_{k}t}\right\|}_{2}^{2}\right\}\\ \text{s.t.}\overset{K}{\underset{k=1}{\sum }}u_{k}=f, \end{array}$$

where K is the number of modes to be decomposed, *δ*(*t*) represents Dirac function,  ^*∗*^means the convolution operator, and {*u*_*k*_} and {*ω*_*k*_} stand for the *k*th intrinsic mode function (IMF) and center frequency after decomposition.

The solution process of this problem is as follows:

(1) Transform the constrained variational problem to a nonconstrained variational problem by introducing the quadratic penalty factor *α* and Lagrange multiplier *λ*(t):
  (11) $$\begin{array}{c} L\left(\left\{u_{k}\right\},\left\{\omega_{k}\right\},\lambda \right)=\alpha \underset{k}{\sum }{\left\|\partial_{t}\left[\left(\partial \left(t\right)+\frac{j}{\pi t}\right){\;}^{*}u_{k}\left(t\right)\right]\right\|}_{2}^{2}+{\left\|f\left(t\right)-\underset{k}{\sum }u_{k}\left(t\right)\right\|}_{2}^{2}+\langle \lambda \left(t\right),f\left(t\right)-\underset{k}{\sum }u_{k}\left(t\right)\rangle . \end{array}$$
(2) Solving the minimization problem of equation (12), alternating direction method of multipliers (ADMM) is adopted to seek the saddle point of the augmented Lagrange expression by alternatively updating *u*_*k*_^*n*+1^, *ω*_*k*_^*n*+1^, and *λ*^*n*+1^, and *u*_*k*_^*n*+1^ can be obtained by
  (12) $$\begin{array}{c} u_{k}^{n+1}=\underset{u_{k}\in X}{\arg\min}\left\{\alpha {\left\|\partial_{t}\left[\left(\delta \left(t\right)+\frac{j}{\pi t}\right){\;}^{*}u_{k}\left(t\right)\right]e^{-j\omega_{k}t}\right\|}_{2}^{2}+{\left\|f\left(t\right)-\underset{i}{\sum }u_{i}\left(t\right)+\frac{\lambda \left(t\right)}{2}\right\|}_{2}^{2}\right\}, \end{array}$$
where *ω*_*k*_ equals to *ω*_*k*_^*n*+1^, and ∑_*i*_*u*_*i*_(*t*) equals to ∑_*i*≠*k*_*u*_*i*_(*t*)^*n*+1^.

Next, transform to frequency domain by Parseval/Plancherel Fourier isometric transform:

(13) $$\begin{array}{c} {\overset{\wedge }{u}}_{k}^{n+1}=\underset{\overset{\wedge }{u_{k}},u_{k}\in X}{\arg\min}\left\{\alpha {\left\|\text{j}\omega \left[\left(1+\mathrm{sgn}\left(\omega +\omega_{k}\right)\right){\overset{\wedge }{u}}_{k}\left(\omega +\omega_{k}\right)\right]\right\|}_{2}^{2}+{\left\|\overset{\wedge }{f}\left(\omega \right)-\underset{i}{\sum }{\overset{\wedge }{u}}_{i}\left(\omega \right)+\frac{\overset{\wedge }{\lambda }\left(\omega \right)}{2}\right\|}_{2}^{2}\right\}. \end{array}$$

Replace *ω* in (13) with *ω* − *ω*_*k*_ and then we can get

(14) $$\begin{array}{c} {\overset{\wedge }{u}}_{k}^{n+1}=\underset{\overset{\wedge }{u_{k}},u_{k}\in X}{\arg\min}\left\{\alpha {\left\|j\left(\omega -\omega_{k}\right)\left[\left(1+\mathrm{sgn}\left(\omega +\omega_{k}\right)\right){\overset{\wedge }{u}}_{k}\left(\omega \right)\right]\right\|}_{2}^{2}+{\left\|\overset{\wedge }{f}\left(\omega \right)-\underset{i}{\sum }{\overset{\wedge }{u}}_{i}\left(\omega \right)+\frac{\overset{\wedge }{\lambda }\left(\omega \right)}{2}\right\|}_{2}^{2}\right\}. \end{array}$$

(14) is then converted to the form of nonnegative frequency interval integral:

(15) $$\begin{array}{c} {\overset{\wedge }{u}}_{k}^{n+1}=\arg\min\left\{\int_{0}^{\infty }4\alpha {\left(\omega -\omega_{k}\right)}^{2}{\left|{\overset{\wedge }{u}}_{k}\left(\omega \right)\right|}^{2}+2{\left|\overset{\wedge }{f}\left(\omega \right)-\underset{i}{\sum }{\overset{\wedge }{u}}_{i}\left(\omega \right)+\frac{\overset{\wedge }{\lambda }\left(\omega \right)}{2}\right|}^{2}d\omega \right\}, \end{array}$$

and set the first item in (15) to zero to obtain the quadratic optimization problem:

(16) $$\begin{array}{c} {\overset{\wedge }{u}}_{k}^{n+1}\left(\omega \right)=\frac{\overset{\wedge }{f}\left(\omega \right)-\sum_{i\neq k}{\overset{\wedge }{u}}_{i}\left(\omega \right)+\overset{\wedge }{\lambda }\left(\omega \right)/2}{1+2\alpha {\left(\omega -\omega_{k}\right)}^{2}}. \end{array}$$

Similarly, the minimization problem of the center frequency can be obtained by converting the center frequency updating problem to frequency domain:

(17) $$\begin{array}{c} \omega_{k}^{n+1}=\frac{\int_{0}^{\infty }\omega {\left|{\overset{\wedge }{u}}_{k}^{n+1}\left(\omega \right)\right|}^{2}d\omega }{\int_{0}^{\infty }{\left|{\overset{\wedge }{u}}_{k}^{n+1}\left(\omega \right)\right|}^{2}d\omega }, \end{array}$$

where ${\overset{\wedge }{u}}_{k}^{n+1}\left(\omega \right)$ is the Wiener filtering of $\overset{\wedge }{f}\left(\omega \right)-\sum_{i\neq k}{\overset{\wedge }{u}}_{i}\left(\omega \right)$, and *ω*_k_^*n*+1^ represents the center of power spectrum.

Also, the learning process of VMD is as follows:

(1) Initialize $\left\{{\overset{\wedge }{u}}_{k}^{1}\right\}$, {*ω*_*k*_^1^}, $\left\{{\overset{\wedge }{\lambda }}^{1}\right\}$ and *n*.
(2) Update *u*_*k*_ and _*ω*_^*k*^ according to equations (16) and (17).
(3) Update *λ* by
  (18) $$\begin{array}{c} {\overset{\wedge }{\lambda }}^{n+1}\left(\omega \right)\leftarrow {\overset{\wedge }{\lambda }}^{n}\left(\omega \right)+\tau \left[\overset{\wedge }{f}\left(\omega \right)-\underset{k}{\sum }\overset{\wedge }{u^{n+1}}\left(\omega \right)\right]. \end{array}$$
(4) For a given discriminant accuracy of *ε* > 0, if $\sum_{k}\left\|{\overset{\wedge }{u}}_{k}^{n+1}\right\|\sum_{k}{\left\|{\overset{\wedge }{u}}_{k}^{n+1}-{\overset{\wedge }{u}}_{k}^{n}\right\|}_{2}^{2}/{\left\|{\overset{\wedge }{u}}_{k}^{n}\right\|}_{2}^{2}<\varepsilon$, stop iteration, otherwise return to step (2).

#### 3.1.2. VMD-Based Denoising Method

The VMD-based denoising method comprises two steps: (a) decompose the vibration signal by VMD. (b) Calculate correlation coefficients of IMFs obtained by VMD for noise filtering and reconstruct the denoised signal. The parameters *α*, *λ*(t), and K of VMD should be set before decomposition, which may affect the results noticeably.

Correlation coefficient is to describe the correlation degree between the original signal Y and its IMFs *X*(*i*), which is defined as

(19) $$\begin{array}{c} \rho_{\text{i}}=\frac{COV\left(X\left(i\right),Y\right)}{\sqrt{D\left(X\left(i\right)\right)}\sqrt{D\left(Y\right)}}. \end{array}$$

The correlation coefficient also offers a means of measuring the degree of noise contained in IMFs. Thus, by selecting the sensitive IMFs according to (20) below [33], we are able to obtain the reconstructed denoised signal:

(20) $$\begin{array}{c} \mu_{\text{i}}=\frac{\max\left(\rho_{i}\right)}{10{\;}^{*}\max\left(\rho_{i}\right)-3}, \end{array}$$

where *μ*_*i*_ is the threshold of the ith IMF. Retain the IMFs of *ρ*_*i*_ < *μ*_*i*_ as sensitive IMFs for signal reconstruction, and remove the unqualified IMFs directly.

### 3.2. Feature Extraction and Selection

#### 3.2.1. Bearing Fault Features

In feature extraction, to reflect the operation conditions of bearings accurately, objectively, and simply, statistical features are extracted from the denoised signals in this study, including 11 time domain statistical features *F*_1_ ~ *F*_11_ and 12 frequency domain statistical features *F*_12_ ~ *F*_23_ shown in Table 1 [34]. For time domain statistical features extracted from raw signals, *F*_1_ and *F*_3_ ~ *F*_5_ reflect the amplitude and energy of vibration in time domain; *F*_1_ and *F*_6_ ~ *F*_11_ present the distribution of the signal in time series. For frequency domain statistical features extracted from FFT spectrums, *F*_12_ shows the vibration energy in frequency domain; *F*_13_ ~ *F*_15_, *F*_17_, and *F*_21_ ~ *F*_23_ stand for the dispersion and concentration degree of the spectrum; *F*_16_ and *F*_18_ ~ *F*_20_ represent the position variation of the main frequency band.

Here, *x*(*n*) is a signal series in time domain, *n* = 1, 2,…, *N*; *N* is the number of data points. *s*(*k*) is a frequency spectrum of signal *x*(*n*), *k* = 1, 2,…, *K*, *K* is the number of spectrum lines, and *f*_*k*_ is the frequency value of the *k*th spectrum line.

#### 3.2.2. Feature Selection Based on PCA

Although the multidomain features obtained above better describe the signals than using time domain or frequency domain features only, there may be feature redundancy, which will affect the diagnostic performance of the model. Considering the lack of labels of samples in clustering fault diagnosis, a commonly used unsupervised feature reduction algorithms principal component analysis (PCA) is adopted in the diagnosis model. The specific steps of PCA are as follows:

Let the multidomain characteristic matrix obtained above be *X*_*n*×*m*_=[*X*_1_, *X*_2_, ⋯, *X*_*m*_], where the number of samples is *m*, and the dimension of features is *n*, then its covariance matrix *C* can be obtained by

(21) $$\begin{array}{c} C=\frac{1}{m}\left(X-\bar{X}\right){\left(X-\bar{X}\right)}^{T}, \end{array}$$

where $\bar{X}$ is a *n* × *m* matrix composed of row vectors of *X*, $\bar{X_{i}}=1/m\sum_{j=1}^{m}x_{ij},i=1,2,\cdots n$.

After that, the eigenvalues and the eigenvectors of the covariance matrix *C* are calculated by

(22) $$\begin{array}{c} \left|C-\lambda I_{n}\right|=0, \end{array}$$

where *λ*_1_, *λ*_2_, ⋯, *λ*_*n*_ are the eigenvalues of *C*, and *P*_1_, *P*_2_, ⋯, *P*_*n*_ are the corresponding eigenvectors of the eigenvalues.

Arrange the eigenvectors according to the magnitude of the corresponding eigenvalues, take the front *k* rows of eigenvectors to form the matrix *P*, and obtain the *k*-dimensional data *Y* by

(23) $$\begin{array}{c} Y=\text{PX}. \end{array}$$

### 3.3. Bearing Fault Diagnosis Model of VMD-Based Denoising and LENN

Based on the above techniques, a bearing fault diagnosis model of VMD-based denoising and LENN is proposed in this paper, including three stages: (a) signal denoising based on VMD and correlation coefficient calculation of IMFs; (b) feature extraction and selection by PCA; (c) clustering fault diagnosis on LENN. The specific diagnostic steps are as follows, which are shown in Figure 6.

1. After signal acquisition, divide the raw signals into some segments of 2048 data points.
2. For the sake of noise reduction, decompose each signal and calculate correlation coefficients and thresholds of IMFs according to equations (19)∼(20). Reconstruct the signals by retaining the sensitive IMFs and removing the IMFs of *ρ*_*i*_ ≥ *μ*_*i*_.
3. Based on the denoised signals, 11 time domain statistical features are extracted from the signals and 12 frequency domain statistical features are extracted from their FFT spectrums according to Table 1.
4. In order to avoid the influence of redundant features on the diagnosis results and improve the diagnostic speed of the model, PCA algorithm is used to obtain low-dimensional fault features for diagnosis.
5. Finally, the proposed LENN algorithm will identify bearing fault conditions by clustering the obtained low-dimensional feature matrix into different clusters and achieve fault diagnosis.

## 4. Experimental Verification

### 4.1. Experiment of LENN Algorithm on Artificial Datasets

In order to verify the clustering effectiveness and stability of the proposed LENN algorithm on imbalanced data, LENN, ENN-2, and three commonly used clustering algorithms, namely, K-means, fuzzy C-means (FCM), and DBSCAN were experimented on three artificial datasets commonly used for clustering testing, which were Flame, Jain and Aggregation. These three datasets are all in two dimensions with different degrees of imbalance, which are summarized in Table 2. From Figure 7 of the real distributions of the datasets, it can be seen that Flame consists of a circle and a semiring, Jain contains two semirings, and Aggregation is composed of many rounded or crescent clusters with two clusters connected, which increase the difficulty of clustering.

Adopt Rand Index to evaluate the clustering results of the algorithms here, which is defined as

(24) $$\begin{array}{c} \text{RI}=\frac{a+b}{a+b+h+g}, \end{array}$$

where *a* denotes the number of data pairs (*x*_*i*_, *x*_*j*_) whose clustering results and real labels are in the same category; *b* represents the number of data pairs (*x*_*i*_, *x*_*j*_) whose clustering results and real labels fall in the different categories; *h* denotes the number of data pairs (*x*_*i*_, *x*_*j*_) whose clustering results are of the same category while real labels are of different categories; and *g* represents the number of data pairs (*x*_*i*_, *x*_*j*_) whose clustering results turn to be of different categories while real labels turn to be of the same category.

In the experimental process of LENN, the optimal value range of *λ* was narrowed in each round of the experiment based on $\left(0\sqrt{\max\left(x_{\text{ij}}\right)}\right]$ to obtain the optimal *λ*, and the optimal *λ* selection processes of LENN on three datasets are shown in Figure 8. As can be seen from the figure, RI reaches a peak at the inflection point of the EDe drop-down curve, and the corresponding value of *λ* is just the desired *λ*, and for ENN-2, the optimal *λ* was determined in the same way based on (0, 1]. The parameter K of K-means was set according to the real number of categories of each experimental dataset, and the parameter setting of FCM was the same as above. In the training process of DBSCAN, the optimal combination of the radius parameter *ε* and the field density threshold MinPts was searched for several times with the initial range of *ε* set as (0, 2] and the initial range of MinPts set as [2, 10]. In order to eliminate the influence of the sample input order on the experimental results, each experiment was conducted for ten times by disrupting the sample input order randomly to obtain RI score of the five algorithms, which are depicted in boxplots in Figure 9 and summarized in Table 3.  Figure 10 presents the clustering performances of LENN graphically on three datasets.

In general, LENN achieved better performances in higher accuracy and stability on the three different datasets. Comparing Figure 9 and Table 3, it can be observed that, in terms of clustering accuracies, LENN and DBSCAN were not affected by the shape of data distribution, showing higher RI scores overall; while ENN-2, K-means, and FCM were highly affected by the shape of data distribution, all of them performed worse on semiorbicular clusters than rounded clusters, among which ENN-2 scored lowest on Flame and FCM scored lowest on Jain; in terms of clustering stability, which was visible in Figure 9, LENN showed extremely stable clustering performances on different input orders of samples, and there were small fluctuations in clustering stability of DBSCAN, K-means, and FCM, while ENN-2 showed the worst stability with the largest range of RI reaching 0.2436 on Flame. In particular, LENN scored highest on both Flame and Jain with nearly no impact of imbalanced data distribution on clustering, while scored slightly lower than that of DBSCAN on Aggregation. That was because, for Flame and Jain in Figure 10, all misclassified points of LENN, which were considered as noise, were individuals far away from their surrounding points; while for Aggregation, two clusters were closely connected distinctly by several data points, resulting in the algorithm which classified the two connected clusters as one cluster because of LENN's iterative distinguish mechanism; in spite of this, LENN could still fully identify the other minority clusters in Aggregation. As for ENN-2, only a small number of cases showed higher clustering accuracies on Aggregation, indicating that ENN-2 is better at processing rounded clusters, but still relies heavily on an appropriate sample input order. It could be concluded that the proposed LENN algorithm could deal with the clustering problem on imbalanced data in terms of higher accuracy and stability, addressing the limitations of dependency on input order of samples.

### 4.2. Bearing Fault Diagnosis Process of Proposed Model

The main purpose of this work was to establish an effective bearing fault diagnosis model on imbalance data with noise, so in this part, experiments were carried out based on bearing fault data from Case Western Reserve University [35, 36] to test the performance of the proposed VMD-based denoising and LENN model by comparing with the ENN-2-based model.

#### 4.2.1. Experimental Data

The test rig for data acquisition is shown in Figure 11, which consists of a motor driving a shaft, a force meter, a torque transducer, and an electrical control device. In this part, we selected the data of a 6205-2RS deep-groove ball bearing from SKF Company, which were grouped into five categories, including normal, minor inner race fault (with the fault size of 0.1778 mm), serious inner race fault (with the fault size of 0.5334 mm), minor ball fault (with the fault size of 0.1778 mm), and serious ball fault (with the fault size of 0.5334 mm). After dividing the raw signals into segments of 2048 data points, five datasets above comprised the whole data of this experiment with the imbalance degree of 2 : 1:1 : 1:1, which are listed in Table 4.

#### 4.2.2. Signal Denoising and Feature Extraction and Selection

Firstly, VMD was carried out on the segmented fault samples. Here, set *α*  = 2000, *λ*(*t*)  = 1.5, and the initial distribution of center frequency was uniform. Considering improper selection of the number of decomposition K will lead to excessive or insufficient decomposition, therefore, K was determined according to the change of the center frequency of each mode in this paper. Taking VMD results of minor inner race fault (MIF) for example, as shown in Table 5, there were similar center frequencies appearing when *K* = 5, which may be attributed to mode mixing and excessive decomposition. Thus, K was set as four. Similarly, the number of decomposition K of other datasets was determined to be four, and the VMD results of a sample of five conditions are shown in Figure 12.

Then, the correlation coefficients and thresholds corresponding respectively to IMFs and the original signal were calculated according to equations (19)∼(20). The obtained results of all samples are graphically presented in Figure 13. Retain the corresponding IMFs whose correlation coefficient is above the red line and get the reconstructed signals.

Next, after signal denoising, extract the 23-dimensional features of each sample from both time and frequency domain according to Table 1, and PCA was used for feature selection and dimension reduction. By comparing the dimensionality reduction results in two and three dimensions in Figure 14, it is visible that, in two dimensions, the cluster of normal is far away from others, while the other four clusters are pretty closer; moreover, the clusters of the same parts with different severities are very close to each other, with connected and overlapped points appearing in the clusters of minor and serious inner race fault, which is not conducive to fault diagnosis. In three dimensions, all the clusters could be well separated, and for the clusters of the same parts with different severities, there seem to be no overlaps among the clusters. Therefore, the feature matrix of three dimensions was selected and finally input into the proposed LENN and ENN-2 algorithms.

#### 4.2.3. Fault Diagnosis Results and Analysis

At the end, the obtained matrix was input into LENN and ENN-2 using RI in (24) for comparison. Similarly, for the sake of eliminating the influence of sample input order on experimental results, each diagnosis experiment was conducted for 10 times by randomly shuffling the input order of samples. Two of the diagnosis results of ENN-2 and LENN-based models are depicted in Figure 15, with the detailed results summarized in Table 6.

It is particularly evident from the results that overall, there was a marked increase in the performance of LENN-based model than that of ENN-2-based model in terms of clustering accuracy and stability. As can be seen from Figure 15, both of the two models performed well on the data of MIF, SIF, MBF, and SBF because of the compact data distribution and good differentiation, with only three SIF points misclassified into MIF in ENN-2-based model. However, for the cluster in normal condition, its distribution was relatively loose, resulting in ENN-2-based model which could not identify the whole cluster correctly and generated multiple clusters and noise points in the results, while LENN-based model only marked very few points at the edge of the cluster as noise which were far from their near points, and from Table 6, it can be observed that ENN-2-based model needed an average iteration of two epochs to converge, while LENN-based model converged in only one epoch, and a significant improvement of RI score was obtained in LENN-based model (0.9754) than ENN-2-based model (0.5835). In addition, the clustering results of ENN-2-based model changed greatly with different sample input orders, while the performances of LENN-based model were very stable. All the results strongly confirm the proposed model preserves higher clustering accuracy and more stable performances.

### 4.3. Impact of Imbalance Degree of Datasets on Diagnostic Models

As outlined in the introduction, the problem of imbalanced data fault diagnosis in real industrial production increases the difficulty of clustering fault diagnosis. Thus, the impact of different imbalance degrees of datasets on diagnostic models was investigated experimentally. The bearing fault data used in Section 4.2 was still adopted in this experiment, and based on the signal denoising and feature extraction and selection method proposed in this paper, four diagnostic models commonly used in clustering diagnosis were constructed and compared on datasets in different imbalance degrees selected randomly by certain proportions (shown in Table 7), which were models on LENN, K-means, FCM, and DBSCAN. The specific parameter settings of the models were in line with the settings in Section 4.1. To evaluate the performances and measure the ability of the models to deal with the clustering problem on imbalanced data, RI, macro-recall, and macro-F score were adopted in this experiment, and by conducting each experiment randomly for 10 times, we were able to get the average scores of each model.

Macro-recall measures the clustering performance of each class, especially the minority classes, which can be computed by

(25) $$\begin{array}{c} \text{macro}-R=\frac{1}{n}\overset{n}{\underset{i=1}{\sum }}\text{Recall}=\frac{1}{n}\overset{n}{\underset{i=1}{\sum }}\frac{{\text{TP}}_{i}}{{\text{TP}}_{i}+{\text{FN}}_{i}}, \end{array}$$

where TP_*i*_ and FN_*i*_ represent the number of correctly and incorrectly predicted samples of the *i*th class, respectively.

Macro-F score is a comprehensive evaluation of the precision and recall of clustering results, which is defined as

(26) $$\begin{array}{c} \text{macro}-F1=\frac{\left(1+\beta^{2}\right)\times \text{macro}-R\times \text{macro}-P}{\beta^{2}\times \left(\text{macro}-R+\text{macro}-p\right)}, \end{array}$$

where *β* denotes the relative importance of macro-R and macro-P, which is usually set as one, and macro-P can be obtained by

(27) $$\begin{array}{c} \text{macro}-P=\frac{1}{n}\overset{n}{\underset{i=1}{\sum }}\text{Precision}=\frac{1}{n}\overset{n}{\underset{i=1}{\sum }}\frac{{\text{TP}}_{i}}{{\text{TP}}_{i}+{\text{FP}}_{i}}, \end{array}$$

where FP_*i*_ represents the number of samples which are misclassified into the ith class but do not belong to that class actually.

Table 8 collects the scores of the models on four datasets in different imbalance degrees. Two extreme cases with data imbalance degrees of 2 : 1 : 1 : 1 : 1 and 10 : 1 : 1 : 1 : 1 are taken to draw confusion matrices of the clustering results, which are shown in Figure 16.

It is apparent that, with the increase of data imbalance degrees, the clustering scores of all models showed a downward trend to varying imbalance degrees on the whole, among which LENN-based model performed noticeably best in all cases, while the configurations of K-means and FCM-based models were far from optimal. Comparing Table 8 and Figure 16, it can be observed that, the proposed model achieved considerably higher scores than other three models on all the datasets. Even on dataset 4 of the most extreme imbalance degree of 10 : 1 : 1 : 1 : 1, LENN-based model also recognized four minority clusters precisely, with ten samples of minor inner race fault, nine samples of serious inner race fault, eight samples of minor ball fault, and nine samples of serious ball fault identified correctly, DBSCAN-based model identified relatively few samples of these minor clusters; while K-means-based model regarded the samples of the same position but different severities as one cluster, failing to further subdivide the severities of samples, and FCM-based model directly identified all the four minority clusters as the same cluster, which scored lowest among the models. In addition, in the training process of LENN-based model on datasets with different imbalance degrees, the value of optimal *λ* grew gradually with the increase of data imbalance degree (shown in Figure 17). This was because, as the samples became more and more sparse, the distances between the samples increased, which required a larger *λ* to construct an extension correlation relationship between the samples, and this also indicated that the value of optimal *λ* was related to the final clustering results. In other words, the smaller of *λ*, the more precise the constructed extension relationship between samples would be, and the higher the accuracy of the proposed model could be obtained.

In conclusion, the imbalance degree of datasets increases the difficulty of fault diagnosis, especially for clustering algorithms relying on the selection of initial center points, and the appearances of minority clusters make it difficult for these algorithms to identify the fault categories correctly by distance calculation. At the same time, surprising outcomes of the experiments manifest that, by expressing the information of minority clusters more precisely through the constructed extension correlation function, the proposed LENN-based model shows good efficiency in identifying the minority clusters on imbalanced data.

## 5. Conclusions

1. A novel clustering algorithm called linked extension neural network (LENN) is developed based on extension neural network-type 2 (ENN-2), which is far less sensitive to initial point selection and sample input order by improved correlation function and new iterative method. Furthermore, to evaluate the clustering performance, extension density is proposed as an evaluation target for this algorithm.
2. With the intention of improving the bearing fault diagnosis ability on imbalanced data with noise, a clustering fault diagnosis model of VMD-based denoising and LENN is constructed. The experimental results provide compelling evidence that the proposed model preserves powerful identification ability of minority fault clusters and achieves better diagnosis performance on imbalanced data with noise.

## Figures and Tables

**Figure 1:** Structure of linked extension neural network (LENN).

**Figure 2:** Image of correlation function ED in ENN-2.

**Figure 3:** Image of new correlation function ED in LENN.

**Figure 4:** Iterative approaches: (a) ENN-2 and (b) LENN.

**Figure 5:** The influence of hyperparameter *λ* on LENN clustering process: (a) a smaller *λ* and (b) a bigger *λ*.

**Figure 6:** Flowchart of the proposed bearing fault diagnosis model.

**Figure 7:** The real distributions of the datasets. (a) Flame. (b) Jain. (c) Aggregation.

**Figure 8:** The optimal selection processes of LENN on three datasets. (a) Flame. (b) Jain. (c) Aggregation.

**Figure 9:** Boxplots of the results of five algorithms on three datasets. (a) Flame. (b) Jain. (c) Aggregation.

**Figure 10:** Clustering performances of LENN on three datasets. (a) Flame. (b) Jain. (c) Aggregation.

**Figure 11:** CWRU bearing test rig35.

**Figure 12:** VMD results of a sample of five conditions: (a) normal, (b) minor inner race fault, (c) serious inner race fault, (d) minor ball fault, and (e) serious ball fault.

**Figure 13:** Results of correlation coefficient and threshold calculation.

**Figure 14:** Dimensionality reduction results of bearing fault data: (a) in two dimensions and (b) in three dimensions.

**Figure 15:** Diagnosis results of the models: (a) ENN-2-based model and (b) LENN-based model.

**Figure 16:** Confusion matrices of the results on two imbalance degrees of the datasets (2 : 1 : 1 : 1 : 1 and 10 : 1 : 1 : 1 : 1): (a) LENN on Dataset 1, (b) K-means on Dataset 1, (c) FCM on Dataset 1, (d) DBSCAN on Dataset 1, (e) LENN on Dataset 4, (f) K-means on Dataset 4, (g) FCM on Dataset 4, and (h) DBSCAN on Dataset 4.

**Figure 17:** RI and optimal *λ* of LENN-based model on data with different imbalance degrees.

**Table 1:** Statistical features of time domain and frequency domain.

No.	Equation
Time domain features	
*F*_1_	∑_1_^*N*^*x*(*n*)/*N*
*F*_2_	$\sqrt{\sum_{1}^{N}\left(x\left(n\right)-F_{1}\right)/N-1}$
*F*_3_	${\left(\sum_{1}^{N}\sqrt{\left|x\left(n\right)\right|}/N\right)}^{2}$
*F*_4_	$\sqrt{{\sum_{1}^{N}\left(x\left(n\right)\right)}^{2}/N}$
*F*_5_	max|*x*(*n*)|
*F*_6_	∑_1_^*N*^(*x*(*n*)−*F*_1_)^3^/(*N* − 1)*F*_2_^3^
*F*_7_	∑_1_^*N*^(*x*(*n*)−*F*_1_)^4^/(*N* − 1)*F*_2_^4^
*F*_8_	*F*_5_/*F*_4_
*F*_9_	*F*_5_/*F*_3_
*F*_10_	*F*_4_/1/*N*∑_1_^*N*^|*x*(*n*)|
*F*_11_	*F*_5_/1/*N*∑_1_^*N*^|*x*(*n*)|
Frequency domain features	
*F*_12_	∑_1_^*K*^*s*(*k*)/*K*
*F*_13_	∑_1_^*K*^(*s*(*k*)−*F*_12_)^2^/*K* − 1
*F*_14_	∑_1_^*K*^(*s*(*k*)−*F*_12_)^4^/*KF*_13_^2^
*F*_15_	$\sum_{1}^{K}{\left(s\left(k\right)-F_{12}\right)}^{3}/K{\left(\sqrt{F_{13}}\right)}^{3}$
*F*_16_	∑_1_^*K*^*f*_*k*_*s*(*k*)/∑_1_^*K*^*s*(*k*)
*F*_17_	$\sqrt{\sum_{1}^{K}{\left(f_{k}-F_{16}\right)}^{2}s\left(k\right)/K}$
*F*_18_	$\sqrt{\sum_{1}^{K}f_{k}^{2}s\left(k\right)/\sum_{1}^{\text{K}}s\left(k\right)}$
*F*_19_	$\sqrt{\sum_{1}^{K}f_{k}^{4}s\left(k\right)/\sum_{1}^{K}f_{k}^{2}s\left(k\right)}$
*F*_20_	$\sum_{1}^{K}f_{k}^{2}s\left(k\right)/\sqrt{\sum_{1}^{K}s\left(k\right)\sum_{1}^{K}f_{k}^{4}s\left(k\right)}$
*F*_21_	*F*_17_/*F*_16_
*F*_22_	∑_1_^*K*^(*f*_*k*_ − *F*_16_)^3^*s*(*k*)/*KF*_17_^3^
*F*_23_	∑_1_^*K*^(*f*_*k*_ − *F*_16_)^4^*s*(*k*)/*KF*_17_^4^

**Table 2:** Description of the artificial datasets.

No.	Dataset	Degrees of imbalance	Feature dimensions	Number of categories	Number of samples
1	Flame	147 : 93	2	2	240
2	Jain	276 : 97	2	2	373
3	Aggregation	272 : 170 : 127 : 105 : 45 : 35 : 34	2	7	788

**Table 3:** RI scores of the five algorithms.

Algorithm	Target	Flame	Jain	Aggregation
LENN	Mean	0.9284	0.9971	0.8061
	Range	0	0	0

ENN-2	Mean	0.3547	0.4941	0.8033
	Range	0.2436	0.0998	0.1240

K-means	Mean	0.4311	0.3217	0.7663
	Range	0	0.0060	0.0024

FCM	Mean	0.4422	0.3004	0.7005
	Range	0	0	0.1276

DBSCAN	Mean	0.9028	0.9584	0.8934
	Range	0.0273	0	0.0003

**Table 4:** Description of bearing fault data.

Fault type	Motor speed (rpm)	Motor load (hp)	Sample frequency (kHz)	Fault size (mm)	Number of samples
Normal (N)	1797	0	12	-	119
Minor inner race fault (MIF)	1797	0	12	0.1778	59
Serious inner race fault (SIF)	1797	0	12	0.5334	59
Minor ball fault (MBF)	1797	0	12	0.1778	59
Serious ball fault (SBF)	1797	0	12	0.5334	59

**Table 5:** Center frequencies corresponding to different values of *K* of minor inner race fault.

*K*	Center frequency (Hz)				
2	693	2776			
3	685	2740	3578		
4	615	1301	2745	3579	
5	615	1300	2729	3345	3616

**Table 6:** Detailed results of ENN-2- and LENN-based models.

Model	Average epochs	Average score	Max score	Min score	Range
ENN-2	2	0.5835	0.6833	0.4520	0.2313
LENN	1	0.9754	0.9754	0.9754	0

**Table 7:** Imbalance degrees of experimental data.

No.	The number of samples in each condition (N : MIF : SIF : MBF : SBF)	Imbalance degree
Dataset 1	100 : 50 : 50 : 50 : 50	2 : 1 : 1 : 1 : 1
Dataset 2	100 : 30 : 30 : 30 : 30	3 : 1 : 1 : 1 : 1
Dataset 3	100 : 20 : 20 : 20 : 20	5 : 1 : 1 : 1 : 1
Dataset 4	100 : 10 : 10 : 10 : 10	10 : 1 : 1 : 1 : 1

**Table 8:** Average scores of models on datasets in different imbalance degrees.

No.	Target	LENN	K-means	FCM	DBSCAN
Dataset 1	RI	0.9485	0.5191	0.5301	0.8278
	Macro-R	0.9700	0.4960	0.4960	0.9140
	Macro-F1	0.9667	0.4933	0.4933	0.9333

Dataset 2	RI	0.9314	0.4806	0.4814	0.8113
	Macro-R	0.9510	0.4950	0.4950	0.8901
	Macro-F1	0.9487	0.4827	0.4827	0.9052

Dataset 3	RI	0.9250	0.4522	0.4376	0.6839
	Macro-R	0.9322	0.4950	0.4950	0.8130
	Macro-F1	0.9367	0.4827	0.4827	0.8486

Dataset 4	RI	0.8920	0.3822	0.2024	0.4329
	Macro-R	0.9100	0.4940	0.4860	0.7500
	Macro-F1	0.9357	0.4786	0.4500	0.8929

## Data Availability

The labeled dataset used to support the findings of this study are available from the corresponding author upon request.
